# *Cordyceps militaris* Carotenoids Protect Human Retinal Endothelial Cells against the Oxidative Injury and Apoptosis Resulting from H_2_O_2_

**DOI:** 10.1155/2022/1259093

**Published:** 2022-09-30

**Authors:** Lin Lan, Shengyu Wang, Shuhua Duan, Xiangyu Zhou, Yufeng Li

**Affiliations:** Molecular Biology Laboratory, College of Food and Biological Engineering, Pidu District, Xihua University, Chengdu City, Sichuan Province, China

## Abstract

Vision loss is primarily caused by age-related macular degeneration (AMD) due to oxidative retinal pigment epithelial (RPE) cell injury. Carotenoid utilization is deemed a possible strategy for treating AMD. *Cordyceps militaris* has advantages like immunomodulatory, anti-inflammatory, and antioxidative characteristics. This paper assessed the possible protective influence of carotenoids obtained by isolating and purifying the *Cordyceps militaris* (CMCT) into human RPE cells (ARPE-19) damaged by hydrogen peroxide (H_2_O_2_). The findings demonstrated that CMCT safeguarded the ARPE-19 cells against the damage and apoptosis caused by H_2_O_2_ and oxidative stress via Bcl-2 protein upregulation, as well as the expression of Bax and cleaved caspase-3 protein. In addition, CMCT treatment increased cell survival and restricted the generation of H_2_O_2_-induced reactive oxygen species (ROS) and the protein expression of NADPH oxidase-1 (NOX1). Additionally, the CMCT treatment of H_2_O_2_-induced ARPE-19 cells ameliorated high malondialdehyde (MDA) levels in oxidative stress-induced cells. The catalase (CAT), superoxide dismutase (SOD), and glutathione peroxidase (GSH) returned to standard levels, which were governed by the higher expression of nuclear Nrf2 protein in the ARPE-19 cells. Moreover, this study showed that CMCT safeguarded the ARPE-19 cells against the damage caused by oxidative stress via its antioxidant activity and antiapoptotic functionality, suggesting the potential therapeutic role of CMCT in AMD prevention and mitigation.

## 1. Introduction

Age-related macular degeneration (AMD) is affected by daily living habits and the environment [1, 2]. It is estimated that up until 2020, AMD has affected 196 million people globally, a number anticipated to rise to 288 million by 2040 [3]. Furthermore, the pathogenesis of AMD is complicated, with no specific therapeutic strategy available. Increasing research demonstrates that injured retinal pigment epithelial (RPE) cells are vulnerable to oxidative stress. Additionally, reactive oxygen species (ROS)-induced RPE, in particular, is considered an initial pathological trigger of AMD occurrence [4–6]. RPE represents a pigment cell layer between the neural retina and the choriocapillaris and is responsible for external retinal protection [7]. These cells display the most active cellular metabolism in ocular tissues and are essential for regenerating and repairing photoreceptor cells, and restricting the retinal entry of toxic plasma and molecules [7].

In addition, oxidative stress produces ROS in cells, causing cell damage and apoptosis [8]. Various clinical studies suggest that damage to RPE cells from prolonged exposure to oxidative stress eventually leads to AMD [9–11]. The RPE cell density decline over time increases the lipofuscin granules, impeding the protective effect against oxidative stress. Consequently, increasing interventions against oxidative stress in RPE cells may provide a therapeutic approach to slow down early AMD progression.

Extensive research data have demonstrated that natural antioxidants derived from plants prevent and ameliorate AMD by protecting RPE cells from oxidative stress injury [12, 13]. Modulating retinal oxidation via daily dietary strategies is vital in slowing or attenuating AMD development. Recent research has indicated that the natural antioxidants found in legumes, plants, vegetables, fruit, and medicinal herbs, including flavonols, penicillin, carotenoids, vitamin E, vitamin C, resveratrol, polyphenols, and curcumin, are effective in reducing functional retinal damage and essential for retinal tissue microcirculation and protecting against oxidative stress changes [14–16]. This suggests that moderately consuming antioxidants via diet daily can help alleviate or delay the occurrence of AMD [17]. Some studies have indicated that specific carotenoids constitute macular pigments and protect the macula from oxidative damage. *Chrysanthemum* contains various natural bioactive components and pharmacological characteristics like antitumor, antioxidative, immunomodulatory, antiaging, and antibacterial activity [18], and is widely used in many Asian countries for medicinal and health purposes. Furthermore, *Cordyceps militaris* primarily consists of carotenoids, ergosterol, adenosine, cordycepin, proteins, ascorbic acid, phenols, and polysaccharides, providing it with unique medicinal properties [19]. In particular, carotenoids exhibit natural immunomodulatory, antioxidative, antitumor, antiaging, and antibacterial properties, as evidenced by several related studies [20]. However, the antioxidative effect of *Cordyceps militaris* carotenoids on RPE cells damaged by hydrogen peroxide remains known. Therefore, this study investigates the protective effect of *Cordyceps militaris* carotenoids on undifferentiated human retinal epithelial cells (ARPE-19) cells to explore their activity against oxidative damage while discussing the possible mechanisms behind this effect.

## 2. Methods and Materials

### 2.1. Test Kits and Reagents

The *Cordyceps militaris* was acquired from the Nanjiang Hongxing Biological Company in Bazhong City (Sichuan Province, China) (Figure 1), while dimethyl sulfoxide (DMSO), Dulbecco's Modified Eagle Medium (DMEM), acetonitrile, and 3-(4,5-dimethylthiazol-2-yl)-2,5-diphenyltetrazolium bromide (MTT), were supplied by Sigma-Aldrich, Inc. in St. Louis (MO, USA). Mitsubishi Chemical Holdings (Japan) provided the HP Macroporous Adsorption Resin, while the Jiancheng Institute of Bioengineering (Nanjing, China) supplied the total capacity test kit, catalase (CAT), malondialdehyde (MDA), superoxide dismutase (SOD), and glutathione (GSH). Biotechnology Hyclone Inc. (Los Angeles, USA) supplied trypsin (0.25%), streptomycin, penicillin, and fetal bovine serum (SV3087), while ALPCO (Salem, NH, USA) provided the annexin V-FITC kit for apoptosis detection. Furthermore, Santa Cruz Biotechnology in Santa Cruz (CA, USA) provided the anti-NADPHoxidase-1 (NOX1), anti-Nrf2, *β*-actin, caspase-3, Bcl-2, and Bax principal antibodies. All additional reagents were provided by Sigma-Aldrich (St. Louis, MO, USA) unless stated to the contrary.

### 2.2. Isolating and Purifying the *Cordyceps militaris* Carotenoids

Fresh *Cordyceps militaris* was subjected to air-drying at 60°C until a steady weight was reached, it was then crushed and sieved. Next, a 2 g sample was mixed with acetone-60% ethanol (2 : 1, v/v) in 20 ml, followed by the addition of 0.5% compound enzymes at pH 4 for 45 min at 50°C. The sample was sonicated for 1.5 h, after which the supernatant was diluted 100 times via centrifugation at 4500 rpm for 10 min to obtain the subsequent *Cordyceps militaris* crude carotenoid extract (CMC).

The CMC samples were purified further via adsorption using an HP-20 macroporous resin column (particle sizes: 0.3–1.2 mm) ≥ 90%, using a 60% ethanol eluent. The eluate was concentrated to a paste at lower pressure (60 rpm, 50°C/min) using a rotary evaporator. The concentrated, dried CMCT was collected and stored at an ultra-low temperature for later use.

### 2.3. Analysis of the Carotenoids and Pigments

The freeze-dried CMCT was dissolved in methanol in an ultrasonic bath, after which a 0.22 *μ*m membrane was used to filter the sample solution while protected from light for carotenoid identification and subjected to ultra-performance liquid chromatography (UPLC). The analysis occurred according to a modified technique delineated before [21]. This process used a Waters C18 reversed-phase column (dimensions: 2.1 × 50 mm and 1.7 *μ*m) at a steady 30°C temperature, 2 *μ*l injection volume, and a flow rate of 0.25 ml/min. The elution process included a pure methanol solution for A, while B comprised a 0.1% formic acid solution. Furthermore, the program consisted of 0 min, 100% A; 4 min, 70% A; 16 min, 45% A; 25∼28 min, 10% A; 32∼40 min, 45% A, at a detection wavelength of 445 nm. High-resolution mass spectrometry conditions: electrospray ion source, positive ion mode, perimeter scan range *m*/*z*: 50–1000, drying temperature: 450°C, capillary voltage: 5500 V, drying gas flow rate: 40 L/min, and DAD detection wavelength range: 380 nm∼600 nm. Fourier transform infrared (FTIR) spectrometry: the CMCT-potassium bromide mixture (2 : 1, v/v) was ground into a powder and pressed into tablets, after which the infrared absorption was detected in a wavelength range of 500–4000 cm^−1^ using the transparent potassium bromide tablets.

### 2.4. Culturing the ARPE-19 Cells

The ARPE-19 cells, provided by the American Type Culture Collection (ATCC), were cultivated in DMEM/F12 supplemented with streptomycin at 100 *μ*g/ml (SV3010 Los Angeles, CA, USA), penicillin at 100 U/ml (Los Angeles, CA, USA), and 10% fetal bovine serum inactivated by heat (Los Angeles, CA, USA) via incubation in 5% CO_2_ at 37°C. After reaching 90% fusion, the cells were passaged every 3–4 d using trypsin at 0.25% (Biotechnology Hyclone Inc., LA, USA) and inoculated into 96-well culture plates for subsequent experiments.

### 2.5. Oxidative Stress Induction Using H_2_O_2_

The ARPE-19 cells were placed on 96-well plates at 1 × 10^5^ cells/well. They were left overnight and allowed to replicate and fuse. DMEM/F12 containing H_2_O_2_ (0–500 *μ*M) was used to culture the cells for 12 h, while cells without H_2_O_2_ served as a control.

### 2.6. MTT Assays

The cell viability was ascertained via the MTT technique. To determine the performance of CMCT against the toxicity caused by H_2_O_2_, 96-well plates were inoculated with the ARPE-19 cells at 1 × 10^5^ cell/well, treated with different CMCT (1–10 *μ*g/ml) and H_2_O_2_ concentrations for 12 h. Next, 20 *μ*L of the MTT (5 mg/ml) was added to each well for a 4 h incubation period at 37°C. The aspiration of the culture solution from each well was followed by the addition of DMSO at 150 *μ*L of DMSO and electric shaking for 10 min. The reaction was terminated via *β*-crystal dissolution. Using a microplate reader, the absorbance of the samples was immediately measured at 490 nm, while three replicates were obtained for each experiment. The results were illustrated as the absorbance value percentage vs. the control, i.e., the absorbance value of the plate wells, divided by the control percentage.

### 2.7. The Analysis of Cell Apoptosis via Annexin and Flow Cytometry

The apoptosis level was analyzed with an annexin V-FITC/PI apoptosis kit as per the instructions of the manufacturer. The ARPE-19 cells were inoculated into the culture plate at 1 × 10^5^ cells/ml and subjected to treatment with and without CMCT, as well as H_2_O_2_ for 12 h. The collected cells were rinsed two times using cold PBS, after which they were resuspended in a new medium and stained at room temperature for 15 min away from light with annexin V-FITC/PI. Then, they were assessed via flow cytometry (BD Bioscience, USA), while a Cell Quest analysis tool (BD Biosciences, Franklin Lakes, NJ, USA) was used to calculate the degree of apoptosis. The results were as follows: normal cells: annexin-V-negative-PI-negative; early apoptotic cells: annexin-V-positive-PI-negative; late apoptotic or necrotic cells: annexin-V-positive-PI-positive. All experiments were repeated three times.

### 2.8. Measurement of the ROS in the Cells

A ROS assay kit was used following the protocols of the manufacturer to detect the ROS levels in the ARPE-19 cells. The DCF-DA fluorescent probe reacted with the ROS produced by cells to form DCF. The collected cells were subjected to a 30 min incubation period using 10 *μ*M of DCFH-DA reagent in darkness at 37°C, after which ice-cold PBS (1 × 10^5^ cells/ml) was used to rinse them twice, followed by resuspension in phosphate buffer. The fluorescence intensity was determined via flow cytometry at respective emission and excitation wavelengths of 525 nm and 488 nm.

### 2.9. Determination of the MDA, GSH, CAT, and SOD Levels

The CMCT impact on the oxidative stress in the ARPE-19 cells was determined after the different treatments, using the SOD, MDA, CAT, and GSH oxidative biomarkers. The ARPE-19 cells were subjected to a 24 h incubation period in 6-well plates (1 × 10^6^ cells/well), followed by applying different CMCT concentrations for 12 h and H_2_O_2_ (400 *μ*g/ml) for 12 h. Next, the collected cells were rinsed two times using ice-cold PBS. The oxidative biomarkers were then measured using the appropriate analytical kits using the protocols of the manufacturers.

### 2.10. Western Blot Analysis

This analysis occurred according to a previously delineated method. Ice-cold PBS was used to wash the ARPE-19 cells twice. The cell lysates were extracted from the collected cells with RIPA lysis buffer, centrifuged at 4°C and 12,000 rpm for 15 min to obtain the supernatant, and measured via a BCA Protein Assay Kit to determine the protein level. Equal quantities of 30 *μ*g of protein were relocated to polyvinyl fluoride (PVDF) membranes along with 12% sodium dodecyl sulfate-polyacrylamide for electrophoretic separation. The samples were exposed for 1 h to 5% skim milk and subjected to overnight incubation at 4°C with the *β*-actin (1 : 1000) Bc1-2 (1 : 200), Bax (1 : 500), caspase-3 (1 : 500), anti-Nrf2 (1 : 300), and NOX1 (1 : 500) primary antibodies. This was followed by room temperature incubation for 2 h using the secondary, horseradish peroxidase-conjugated antimouse antibody (1 : 2000). After repeatedly rinsing with PBST, the individual protein expression was observed via an ECL western blotting assay test kit as per the prescribed procedure.

### 2.11. Statistical Evaluation

All experiments were performed at least three times, and the data after experiments were expressed as mean ± standard deviation (SD). Statistical analysis was performed using GraphPad Prism software. Data were analyzed by one-way ANOVA. *P* < 0.05 was considered significant.

## 3. Results

### 3.1. CMCT Preparation and Characterization

The CMCTs were produced using a technique previously described with some modifications [22]. The CMCTs were obtained via crushing, acetone, and ethanol mixed solution extraction and complex enzyme precipitation at an extraction rate of 3888.34 *μ*g/g. Chrysin carotenoids are intracellular pigments. The cell walls were disrupted and extracted with cellulase and pectinase (extraction ratio of 2 : 1), after which the CMC extract was dissolved using acetone and a 60% ethanol solution. ELISA was employed for absorbance determination at 445 nm (Figure 2(a)). The standard curve was configured as *Y* = 0.1093*x* + 0.0801 and *R*2 = 0.9992 (*Y* denoted the absorbance, while *X* signified the pigment level). The macroporous adsorbent resin was used to further separate the CMC, increasing the carotenoid purity for subsequent cellular experiments to 66.24% (Figure 2(b)). Then, the CMCTs were exposed to concentrated sulfuric acid to obtain a blue-green color. Furthermore, exposure to an antimony trichloride chloroform solution yielded a green color, while the color values were consistent with those of olefin carotenoids. Spectroscopic and mass spectrometric analyses confirmed that the pigment purification exhibited general carotenoid characteristics. Five main pigment components were isolated, as shown in (Figure 2(c)). The exact mass numbers were determined from 1 to5 in positive ion [M + H]^+^ mode, yielding values *m*/*z* 629.1862, *m*/*z* 525.4265, *m*/*z* 495.3362, *m*/*z* 523.2778, and *m*/*z* 537.1624. The absorption peaks of the five carotenoids displayed identical absorption spectra and conjugation systems, which were consistent with the essential carotenoid characteristics. Therefore, they are compatible with the basic attributes of carotenoids.

### 3.2. The Influence of CMCT Treatment on the ARPE-19 Cells

The CMCT influence on cell survival was investigated via an MTT assay and presented as the survival rate of the untreated control samples. A slight increase in cell viability increase was evident in the cells subjected to different CMCT treatments at concentrations in a range from 1 *μ*g/ml to 2.5 *μ*g/ml (Figure 3(a)). However, the cell viability declined significantly after exposure to 5 *μ*g/ml CMCT, while a 10 *μ*g/ml CMCT concentration decreased the cell survival rate to 79% in comparison with the untreated samples (*P* > 0.05). Consequently, 1 *μ*g/ml and 2.5 *μ*g/ml CMCT concentrations were utilized for the subsequent experiments. To determine the correct H_2_O_2_ concentration for assessing the impact of CMCT on the cytotoxicity of H_2_O_2_, the ARPE-19 cell viability was examined after 12 h of exposure to H_2_O_2_ (0–500 *μ*M). The cell viability decreased dose-dependently from 100 ± 3.6% in the untreated group to 91.1 ± 1.94% at 50 *μ*M, 78.76 ± 3.3% at 100 *μ*M, 69.1 ± 2.9% at 200 *μ*M, 63.5 ± 2.48% at 250 *μ*M, 41.6 ± 1.85% at 400 *μ*M, and 35.2 ± 1.3% at 500 *μ*M, respectively (Figure 3(b)). Therefore, an H_2_O_2_ concentration of 400 *μ*M was used during the experiments.

This study investigated if the target CMCT safeguarded ARPE-19 cells from destruction by H_2_O_2_. The cells were precultured for 12 h and 24 h in a medium containing CMCT (1 *μ*g/ml, 2.5 *μ*g/ml), which was changed to a new medium containing H_2_O_2_ (400 *μ*M), followed by culturing for 12 h. The results showed significant protection against H_2_O_2_-induced AEPE-19 cell death after 12 h CMCT treatment (1 *μ*g/ml, 2.5 *μ*g/ml) (*P* < 0.05). However, although 24 h CMCT treatment (2.5 *μ*g/ml, 1 *μ*g/ml) displayed only a slight protective effect, no substantial differences were apparent from the control group (*P* > 0.05). Some toxicity was evident in the cells after prolonged pretreatment. Therefore, a 12 h incubation period was selected to assess CMCT protection against H_2_O_2_ damage in the ARPE-19 cells. As illustrated in (Figure 3(c)), pretreatment with 2.5 *μ*g/ml and 1 *μ*g/ml CMCT significantly increased cell viability to 75.6 ± 4.7% and 69.4 ± 6.5%, respectively, displaying substantial variation from the control samples (*P* < 0.05).

### 3.3. CMCT Protection against the RPE Cell Death Caused by H_2_O_2_

RPE cell damage is usually due to oxidative stress. The ability of CMCT to protect against the ARPE-19 cell death caused by H_2_O_2_ was examined by incubating the cells at 1 *μ*g/ml and 2.5 *μ*g/ml CMCT concentrations for 12 h, followed by H_2_O_2_ for 12 h, after which they were observed via phase-contrast microscopy, as shown in (Figure 4(a)). The population dispersion of the stained annexin V-positive cells is demonstrated in (Figure 4(b)). H_2_O_2_ (400 *μ*M) treatment for 12 h significantly increased the apoptotic cell proportion to 63.87 ± 1.7% compared with the control group (5.16 ± 0.34%). However, CMCT (1 *μ*g/ml and 2.5 *μ*g/ml) pretreatment and H_2_O_2_ exposure for 12 h significantly decreased the apoptosis induced by H_2_O_2_ (27.21 ± 1.78% and 38.84 ± 1.58%, *P* < 0.05), when compared to the control cells (3.10 ± 0.67%).

### 3.4. The Impact of CMCT Treatment on the Production of Intracellular ROS and Expression of NOX1 Proteins in the ARPE-19 Cells

Research has shown that the production of ROS exceeds the in vivo clearance limit due to oxidative stress. The subsequent imbalance in the oxidative and antioxidant systems leads to functional and morphological damage in the ganglion, endothelial, and RPE cells [23]. Therefore, this study investigated whether CMCT affected the ROS levels in the ARPE-19 cells after stress. The cells were exposed to different CMCT concentrations (1 *μ*g/ml, 2.5 *μ*g/ml), as well as H_2_O_2_ (400 *μ*M) for 12 h, respectively, after which the ROS levels were measured directly via DCFH-DA staining. H_2_O_2_ significantly elevated the production of intracellular ROS compared to the untreated samples (Figure 5(a)). However, CMCT (2.5 *μ*g/ml, 1 *μ*g/ml) treatment for 12 h significantly reduced the upregulated ROS activity induced by H_2_O_2_ (400 *μ*M). According to (Figure 5(b)), pretreatment with different CMCT concentrations (2.5 *μ*g/ml, 1 *μ*g/ml) attenuated the NOX1 protein expression induced by H_2_O_2_ oxidative stress. Furthermore, some of the differences from the H_2_O_2_ control were statistically significant (*P* < 0.01 or *P* < 0.05).

### 3.5. The Influence of CMCT on Regulating the Antioxidant Content of the ARPE-19 Cells Exposed to H_2_O_2_

Since oxidative stress is crucial in the senescence state of normal ARPE-19 cells, this study examined the activity of MDA, an indicator of lipid oxidation, and GSH, CAT, and SOD, biomarkers of oxidative in the ARPE-19 cells subjected to various treatments. Compared with the untreated cells, H_2_O_2_ pretreatment alone for 12 h yielded higher MDA levels but decreased the GSH, CAT, and SOD activity (Figures 6(a)–6(d)). CMCT treatment alone did not affect the MDA level and three oxidative stress biomarkers. However, after incubation with CMCT (2.5 *μ*g/ml, 1 *μ*g/ml) for 12 h, the MDA level decreased according to the concentration, while the SOD, CAT, and GSH activity wer restored to normal levels. The cellular response to oxidative stress is regulated by Nrf2 to maintain redox homeostasis. It can mitigate the ROS and electrophile damage in cells by inducing and controlling antioxidant protein expression to stabilize the cells and facilitate the dynamic redox balance of the organism. This study assessed the impact of CMCT on the nuclear translocation expression of Nrf2 proteins in the ARPE-19 cells, while observing the upregulation of Nrf2 protein epitope expression after treatment with different CMCT concentrations (1 *μ*g/ml, 2.5 *μ*g/ml) (Figure 6(e)).

### 3.6. The Influence of CMCT on the Protein Expression Associated with ARPE-19 Cell Apoptosis after H_2_O_2_ Exposure

Apoptosis and cell damage are often the result of oxidative stress. Therefore, this study explored whether CMCT effectively protected ARPE-19 cells against apoptosis and assessed the impact of CMCT on the expression of proteins associated with apoptosis. The results of the protein blot analysis are presented in (Figure 7). The ARPE-19 cells subjected to H_2_O_2_ (400 *μ*M) treatment for 12 h showed significantly higher downregulation in the protein expression of Bcl-2, as well as higher cleaved caspase-3 and Bax expression levels than the control group, which was consistent with the flow cytometry results. Moreover, CMCT (1 *μ*g/ml, 2.5 *μ*g/ml) pretreatment for 12 h dose-dependently reversed this, increasing the protein expression of Bcl-2 and significantly decreasing these levels in cleaved caspase-3 and Bax.

## 4. Discussion

Oxidative stress causes apoptosis in retinal endothelial cells. Excess ROS usually generates oxidative stress, leading to intracellular mitochondrial dysfunction and antioxidant system damage, ultimately causing degenerative diseases of the human retinal epithelium, such as AMD [24, 25]. Oxidative stress is primarily caused by the discrepancy between biological scavenging ability and active free radical generation. Fat accumulation, nucleic acid molecule cleavage mutations, protein inactivation and degradation, and photosensitive cell regeneration and repair decline in conjunction with environmental changes and increased age [26]. Consequently, reducing the cellular oxidative stress is critical for slowing AMD progression and facilitating potential treatment options for vision loss.

Clinical trials and research data have shown that the consumption of lutein, vitamins E and C, flavonoids, anthocyanins, zeaxanthin, and carotenoids can enhance cells and strengthen the antioxidant system to maintain good retinal function [27–31]. The minimal level of toxicity and powerful antioxidant capacity of the carotenoids found in natural plants have attracted considerable attention from researchers, rendering them effective as potential therapeutic agents. Singlet oxygen is quenched by carotenoids, scavenging free radicals to restrict lipid peroxidation reactions in vivo and blue light filtering, modulating light stress recovery time and neural processing speed [32]. Functions, Cordyceps militaris, as reported to contain many essential components required by the body, especially CMCT, has high antioxidant efficiency. As far as is known, this study is the first involving the antioxidant impact of CMCT on RPE cells. However, the mechanism underlying its anti-H_2_O_2_-induced oxidative stress effect remains unclear. Therefore, this research investigated the possible effect of CMCT in protecting against the death of retinal endothelial cells caused by H_2_O_2_.

Several studies have shown that H_2_O_2_ exposure induces ROS production while accelerating cell damage and apoptosis [33]. Since RPE cells are located behind photoreceptor cells and are mainly responsible for scavenging the oxidants generated by photoreceptor conversion, ARPE-19 cellular oxidative stress is used as a typical in vitro model to examine the functionality of human RPE cells. This study also revealed the pathogenesis of AMD by inducing oxidative stress and cellular damage [34]. The survival rate of the ARPE-19 cell exposed to 400 *μ*M H_2_O_2_ decreased, while CMCT pretreatment (2.5 *μ*g/ml, 1 *μ*g/ml) substantially restricted the cytotoxicity caused by H_2_O_2_ and increased cell survival while reducing oxidative stress-induced apoptosis. Reports have indicated that protein restricts Bcl-2 and Bax. The increased protein expression of Bax and Bcl-2 alters the permeability of cellular mitochondrial membranes, subsequently inhibiting mitochondrial disruption and prompting the release of cytosolic *c* and cystathionine activation [35]. Moreover, caspase-3 selectively and efficiently cleaves proteins in various signal transduction pathways and is essential for controlling programmed cell death. Bcl-2 overexpression reportedly increases the survival of cells exposed to H_2_O_2_ [36]. The present study indicated that ARPE-19 cell exposure to H_2_O_2_ upregulated the caspase-3 and Bax protein expression. However, Bcl-2 protein expression was downregulated compared to the untreated control groups. H_2_O_2_ exposure elevated the expression of caspase-3 and Bax protein receptors and reduced that of Bcl-2. However, 12 h of CMCT pretreatment (1 *μ*g/ml, 2.5 *μ*g/ml) prior to H_2_O_2_ exposure successfully reversed this, decreasing the protein expression of caspase-3 and Bax, while enhancing that of Bcl-2. This suggests that the ROS generation in the ARPE-19 cells is associated with H_2_O_2_-induced apoptosis. CMCT protects against the ARPE-19 cell damage caused by H_2_O_2_ by inhibiting apoptosis.

ROS generation is associated with the co-interaction between nanoparticles and redox proteins such as mitochondria and NOX1, and cell surface receptors [37]. NOX1 is reportedly a vital enzymatic regulator of redox reactions in vivo and an identified system for ROS production. As one of the primary sources of ROS, NOX1 is crucial for the formation of RPE cell lesions in humans [38]. In addition, the GSH, CAT, and SOD activity, MDA levels, and NOX1 protein expression were examined. This study showed that exposing ARPE-19 cells to H_2_O_2_ significantly decreased the SOD, CAT, and GSH levels, while substantially increasing ROS and MDA production and NOX1 protein expression. However, CMCT treatment reversed these effects. Previous research indicated that the retinal cell apoptosis caused by oxidative stress was responsible for AMD pathogenesis, while the nuclear transcription factor, Nrf2, is crucial for oxidative stress regulation [39]. Nrf2 can upregulate antioxidant enzyme expression, scavenge free radicals, reduce intracellular oxidative stress levels, and decrease cell degeneration. It can also protect cells from oxidative damage by inducing ROS detoxification enzymes [40]. Moreover, Nrf2 is considered one of the most critical intracellular antioxidative stress mechanisms and plays a vital role in AMD treatment [41]. Therefore, the impact of CMCT on the translocation of Nrf2 in the ARPE-19 cells was examined via Western blotting, indicating that the Nrf2 expression was upregulated after CMCT treatment. Furthermore, it highlighted the potential of CMCT to safeguard RPE cells against the oxidative stress resulting from H_2_O_2_ by controlling NOX1 protein expression to reduce the ROS and MDA levels. Contrarily, the nuclear activation of Nrf2 protein increased the antioxidant enzyme activity of SOD, CAT, and GSH. Studies have shown that oxidative stress can reduce cell apoptosis, increase the total amount of apoptosis and ROS production, and prevent cells from oxidative stress-induced damage [42].

Therefore, this study shows that CMCT treatment successfully safeguards ARPE-19 cells against the oxidative damage resulting from exposure to H_2_O_2_ by inhibiting apoptosis, regulating ROS production and MDA formation, and increasing the activity of antioxidant enzymes. It also provides new insight into the ability of CMCT to help forestall and mitigate ocular diseases like AMD. Future research should explore the in vivo preventative and therapeutic effect of CMCT in AMD disease models to determine its complete mechanisms.

## Figures and Tables

**Figure 1:** *Cordyceps militaris* samples.

**Figure 2:** Isolating and purifying *Cordyceps militaris*. (a) A spectrum image of the *Cordyceps militaris* carotenoid extraction solution with three characteristic absorption peaks evident at 420 nm, 445 nm, and 475 nm, the most prominent of which is apparent at 445 nm. (b) Macroporous resin activation. (c) The UPLC chromatogram of the carotenoids identified in *Cordyceps militaris*.

**Figure 3:** The CMCT treatment impact on the ARPE-19 cells. (a) Treatment with different CMCT concentrations (0–10 *μ*g/ml) for 12 h (b) Treatment with different H_2_O_2_ concentrations (0–500 *μ*M) for 12 h (c) Pretreatment with different CMCT concentrations (0–100 *μ*g/ml) and H_2_O_2_ (400 *μ*M) for 12 h, respectively. The information is shown as mean ± SD for three separate replicates. Compared to the control samples: ^*∗*^*P* < 0.05 and ^*∗∗*^*P* < 0.01. Compared to the H_2_O_2_ control samples: ^#^*P* < 0.05 and ^##^*P* < 0.01 Compared to the H_2_O_2_ group: ^##^*P* < 0.01.

**Figure 4:** The CMCT protective impact against the RPE cell death caused by H_2_O_2_. (a) Images of the ARPE-19 cell morphology after CMCT treatment. (b) The influence of CMCT treatment on the apoptosis in the ARPE-19 cells caused by H_2_O_2_ was assessed via flow cytometry and annexin V-FITC/PI. The information is presented as mean ± SD for three separate replicates. Compared to the control group: ^*∗*^*P* < 0.05 and ^*∗∗*^*P* < 0.01. Compared to the H_2_O_2_ control samples: ^#^*P* < 0.05 and ^##^*P* < 0.01.

**Figure 5:** The influence of CMCT treatment on ROS generation and the protein expression of NOX1 in the ARPE-19 cells. (a) The influence of CMCT treatment on the production of ROS caused by H_2_O_2_. (b) The impact of CMCT (1 *μ*g/ml and 2.5 *μ*g/ml) on the protein expression of NOX1 in the ARPE-19 cells after H_2_O_2_ treatment was assayed via flow cytometry. The information is presented as mean ± SD for three separate replicates. Compared with the control group: ^*∗*^*P* < 0.05 and ^*∗∗*^*P* < 0.01. Compared with the H_2_O_2_ control samples: ^#^*P* < 0.05 and ^##^*P* < 0.01.

**Figure 6:** The antioxidant activity in the ARPE-19 cells exposed to H_2_O_2_ is down-modulated by CMCT. (a) The CMCT (1 *μ*g/ml, 2.5 *μ*g/ml) impact on the MDA degradation by lipid peroxide in the ARPE-19 cells after H_2_O_2_ treatment. (b) The CMCT (1 *μ*g/ml and 2.5 *μ*g/ml) impact on the SOD behavior in the ARPE-19 cells after H_2_O_2_ treatment. (c) The CMCT (1 *μ*g/ml, 2.5 *μ*g/ml) impact on the CAT levels in ARPE-19 cells after H_2_O_2_ exposure. (d) The CMCT (1 *μ*g/ml, 2.5 *μ*g/ml) impact on the GSH content in the ARPE-19 cells after H_2_O_2_ exposure. (e) CMCT encourages H_2_O_2_ to down-modulate the degree of intracellular antioxidant levels in ARPE-19 cells. The data are shown as mean ± SD for three separate replicates. Compared with the control group: ^*∗*^*P* < 0.05 and ^*∗∗*^*P* < 0.01. Compared with the H_2_O_2_ control samples: ^#^*P* < 0.05 and ^##^*P* < 0.01.

**Figure 7:** The impact of CMCT treatment on the expression of proteins associated with ARPE-19 cell apoptosis after H_2_O_2_ exposure. (a) The cells received a 12 h CMCT pretreatment at different concentrations (0–10 *μ*g/ml), and H_2_O_2_ (400 *μ*M) treatment for 12 h to examine the changes in the intracellular ROS levels. (b) Flow cytometry was used to analyze the expression of NOX1 proteins in the ARPE-19 cells following exposure to H_2_O_2_ and CMCT (2.5 *μ*g/ml, 1 *μ*g/ml). The data are shown as mean ± SD for three separate replicates. Compared to the control group: ^*∗*^*P* < 0.05 and ^*∗∗*^*P* < 0.01. Compared to the H_2_O_2_ control samples: ^#^*P* < 0.05 and ^##^*P* < 0.01.

## Data Availability

The data supporting the findings of this study are available on reasonable request from the corresponding author.
